The article "Design Model of Cultural and Creative Products Using User Perception Demand Mining" was retracted in 2023. Reasons: suspected computer-generated content; unreliable results or conclusions; concerns about the data; concerns about the results or conclusions.

# Design Model of Cultural and Creative Products Using User Perception Demand Mining

**DOI:** 10.1155/2022/6339184

**Published:** 2022-08-21

**Authors:** Huahua Yang

**Affiliations:** School of Art, Yulin University of Shaanxi Province, Yulin 719000, China

## Abstract

People are becoming more and more aware of the value of design throughout a product's entire life cycle as a result of the fierce competition for industrial products that exists today. The life of a product involves its design, manufacture, sale, and use, and how well these links are managed determines the product's positioning in terms of value in the eyes of consumers. The key to the functional integration of the design is monitoring the entire process and applying the user's emotional needs. A useful tool for assessing users' emotional needs is the perceptual image of a product. An artificial intelligence-driven method for product perceptual design is proposed, and its efficacy is demonstrated by the design of an optometer. This method addresses the issues of incomplete measurement and insufficient sample collection in the traditional users' perceptual cognition measurement. The findings demonstrate that extracting users' perceptual cognition through text mining can assist designers in better understanding users' perceptual needs, resulting in designed products that are more likely to meet users' expectations for satisfaction. A design approach that can increase users' psychological acceptance of products and boost their competitiveness is the perceptual design method, which combines human and artificial intelligence.

## 1. Introduction

People in China are gradually realizing the importance of industrial design in promoting the creation, and the use of industrial products as industrial ingenuity is given more and more attention [1]. The consumer market for goods has now gradually shifted from being enterprise-oriented to being user-oriented. The desire for products to reflect their own cultural preferences, aesthetics, and values is a major driving force behind consumer product purchases, which brings the relationship between culture and design closer and closer [2]. The results of users' perceptual and cognitive analysis of products can be converted into design information and used to create design specifications in contemporary design. These design specifications can help designers create goods that satisfy users' perceptual needs, improving the competitiveness of their offerings [3]. Kansei Engineering is the field that uses user perceptual cognition the most for research and application.

In order to encourage the high-quality development of China's cultural and creative industries, China established the China Beijing International Cultural and Creative Industry Expo in 2006 [4]. Since that time, cultural and creative products have slowly taken over the domestic market for product design, and an increasing number of designers have started to consider and reflect on their own culture in an effort to turn it into creativity and create cultural and creative products that have local recognition [5]. The early stages of Wenchuang product design saw designers deduce and reorganize the extracted cultural symbols and apply them to product design. They realized that the creative source of Wenchuang products could be extracted from the physical modeling involved in traditional culture. Once upon a time, this innovative approach was well received and developed into one of the primary design approaches for Wenchuang products [6]. The typical platform users are identified through research on the current state of the cultural and creative market and the industry's participants. Regular consumers, creative consumers, designers, craftspeople, and manufacturers conduct user interviews and create questionnaires after learning the basic requirements of typical users. To summarize the various needs and relationship statuses of typical users on the platform, as well as the anticipated needs of each typical user on the platform, quantitative research on typical users is conducted [7]. Therefore, applying cultural traits to product design is becoming increasingly important in the fiercely competitive global product market, and higher standards are being placed on the interpretation, extraction, and application of cultural elements in the design process [8].

The article "Design Model of Cultural and Creative Products Using User Perception Demand Mining" was retracted in 2023. Reasons: suspected computer-generated content; unreliable results or conclusions; concerns about the data; concerns about the results or conclusions.

In recent years, with the development of China's culture and design service-related industries, it not only provides people with high-quality cultural and creative products and services but also promotes the innovation and optimization of the cultural industry and the continuous promotion of research on cultural and creative product design [9]. At present, the domestic research on cultural and creative product design mainly focuses on several aspects: The first, starting from the cultural symbols of the target ethnic groups and their visual forms of expression, is to extract representative cultural elements and apply them to modern product design. The second is to explore consumers' cognitive law of the cultural images of the target ethnic groups and transform users' perception and evaluation trend of cultural images into design elements so as to improve the efficiency of cultural and creative product design and users' cultural identity [10]. The third is to analyze the use situation of the target cultural samples as a whole and establish a product design mode driven by cultural connotation, so that cultural elements can be reasonably applied to the design of cultural and creative products. This paper will select the purple teapot as a cultural sample, use the cultural ergonomics theory to sort out its development history and cultural context, summarize the three levels of cultural and creative product design related to the purple teapot, and study the user's subjective modeling preference of the purple teapot based on the perceptual engineering method and eye-tracking technology, so as to obtain the user's visual attention preference, subjective image preference, and beauty preference. Combined with the requirements of cultural sustainable development of purple clay teapots, this paper puts forward the design strategy of cultural and creative products that combines the cultural ergonomic situation with users' subjective preferences and applies it to the design practice of related cultural and creative products. The narrative design elements of creative products are separated into “shape” design elements and “state” design elements. The key design elements of product “shape” and “state” are extracted by qualitative and quantitative methods, and the relationship model between consumers' perceptual images and design elements is constructed by the cluster modeling method in perceptual engineering.

The article "Design Model of Cultural and Creative Products Using User Perception Demand Mining" was retracted in 2023. Reasons: suspected computer-generated content; unreliable results or conclusions; concerns about the data; concerns about the results or conclusions.

Therefore, the goal of this project is to improve the degree of fit and matching between product imagery and user imagery, solve the challenges faced in the process of narrative design, and better support designers in developing products that satisfy users' needs. For psychological feelings in cultural images, beginning with the narrative theme-subtopic-topic element in narrative design theory, the narrative subtopic is divided into image-narrative subtopic and cultural narrative subtopic by synthesizing perceptual image research methods. Second, using the composition theory of narrative design elements, the design components required to create product images are divided into product “form” and product “state” design components, and the related narrative themes are matched through design requirements. The Miao cultural and creative product nightlight is used as an example for practical research, and a product narrative design model based on consumers' perceptual images is created on the basis of the perceptual clustering model to ensure that the images created by the product form do not break away from consumers' psychological cognition.

## 2. Related Work

“Kansei Engineering” is a comprehensive interdisciplinary subject involving arts, humanities, engineering, and other disciplines. Japan Kansei Engineering Society was founded in 1997. Since 2000, the Japan Kansei Engineering Society has held regular annual discussions, where scholars from all over the world can publish their research achievements on Kansei Engineering. Throughout the course of the development of the discipline, early research on the perceptual aspect appeared in the German philosopher G·A·Baumgarten's book “Aesthetic.” The process of text data mining mainly includes text data collection, data preprocessing, text feature mining, and result display. This research has a profound influence on the formation of Kansei Engineering. Combined with the development trend of industrial design, the perceptual design method of products driven by artificial intelligence is put forward.

The article "Design Model of Cultural and Creative Products Using User Perception Demand Mining" was retracted in 2023. Reasons: suspected computer-generated content; unreliable results or conclusions; concerns about the data; concerns about the results or conclusions.

Theien et al. believe that when a good promotion relationship is formed between urban development and urban culture, the two will get better and more stable development and form the unique cultural competitiveness of the city [11]. Zong believes that the cultural and creative industries will lead to the characteristics of low energy consumption and high output to create huge value for the Chinese economy and will become the most competitive industry in the 21st century [12]. Liu and Zhu believe that it is necessary to integrate the cultural and creative value chain to enhance the core competitiveness; build cultural industry clusters to improve the effect of agglomeration development; realize the integration and interaction of cultural creativity to promote the upgrading of industrial structure and the transformation of economic development mode, so as to cope with the opportunities and challenges brought by the cultural creative industry [13]. Li et al. put forward the three-level theory of user's emotion, explored the origin of the user's perceptual image from the cognitive level, and provided a theoretical basis for the subsequent research on product perceptual image [14]. In Sensible Design, Li and Lin pointed out that when consumers describe the perceptual images of products, they tend to use adjectives, such as “exquisite” and “unique,” to describe their feelings about products. Because consumers' individual cognition is different, the perceptual image words they choose to describe are not the same. Therefore, it is necessary to collect users' image needs through semantic differences, questionnaires, and interviews and locate users' perceptual images with data mining methods [15]. Bao and Huang used adjectives to represent users' perceptual image needs and used statistical methods such as factor analysis and cluster analysis to prioritize adjectives to obtain target images that can reflect users' perceptual needs [16]. Chen et al. believe that users have their own tacit knowledge in the perception of product perceptual imagery. This tacit knowledge is extremely critical to the construction of the core competitive advantage of products. Before developing products, designers should make full use of the user's explicit knowledge. In order to understand sexual knowledge, it is also necessary to dig deep into the implicit emotional response related to perceptual cognition in the user's heart [17]. Landoni et al. found that there is a large amount of tacit knowledge in the process of user cognition, which is not easy to accumulate and spread quickly in a short time and has the characteristics of context, culture, and hierarchy [18]. Ho et al. believe that “culture” is the communication channel between the object and the subject, and this communication requires the gravity and inertia of the cultural memory field, which depend on the traction of tacit knowledge [19].

The article "Design Model of Cultural and Creative Products Using User Perception Demand Mining" was retracted in 2023. Reasons: suspected computer-generated content; unreliable results or conclusions; concerns about the data; concerns about the results or conclusions.

In conclusion, it has been discovered through research on perceptual image theory, perceptual image cognition, and product cultural image that consumers have some subjectivity in the actual product image and that their cognition of the product image is highly correlated with their cultural background and life experiences. This research introduces narrative design on the basis of perceptual engineering in order to better design the image of product culture. Its goal is to guide designers in the systematic and scientific conversion of culture into creativity.

## 3. Methodology

### 3.1. Perceptual Cognition Based on Mining Users' Perceptual Needs

Compared with traditional engineering, the most differentiated research in Kansei Engineering is the research on users' “sensibility.” Professor Nagamachi Mitsuo believes that sensibility is a kind of use of sight, hearing, feeling, smell, taste, recognition, balance, and so on. A personal subjective impression is obtained from some artifact or environment. In this process, calculating with the help of psychological, ergonomic, medical, or engineering methods is a discipline that transforms perceptual cognition into design parameters and specifications and is also a way to improve people's pursuit of happiness and emotional satisfaction in the quality of life science.

#### 3.1.1. AI-Driven Approach to Product Perceptual Design

AI-driven approach is as follows: (1) determination of target products and user groups; (2) collection of user perceptual cognition data, which can be collected through user comments, literature, image data, and so on; (3) statistics, classification, and perceptual feature screening of user perceptual cognition information; the methods used include natural language learning (NLP) and computer word computing (CWW) for text mining; (4) mapping the relationship between perceptual features and product attributes, finding the perceptual features corresponding to the physical attributes of the product, and forming the design direction guidance; (5) design realization under the satisfaction of perceptual requirements, including the expansion of designer's thinking and computer-aided calculation and design realization, such as genetic algorithm (GA), deep convolution countermeasure network (dcgan), and pro/engineer-aided design; (6) evaluation and prediction of design scheme, including TOPSIS, AHP, and Bayesian network; (7) optimization and determination of the design scheme and feeding back the information to the starting level to update the perceptual knowledge.

The article "Design Model of Cultural and Creative Products Using User Perception Demand Mining" was retracted in 2023. Reasons: suspected computer-generated content; unreliable results or conclusions; concerns about the data; concerns about the results or conclusions.

#### 3.1.2. Calculation Process of Data Mining Algorithm

The calculation process of the data mining algorithm is as follows: (1) Text data collection: determining the data source and obtaining the corpus are generally the first steps of text data mining. Currently, the required data is usually obtained by grabbing network data. (2) Data preprocessing: due to the huge number of online comments and unstructured data, the comment data collected by web crawler technology can generally meet the requirements of quantity and topic relevance but cannot make the initial data machine readable. (3) Text feature mining: this is the main link in the process of data mining. By using neural network, machine learning [20], data analysis, and other related technologies, we can mine the key elements such as product features, comment views, and user emotions hidden in the comment text and realize the classification, clustering, association analysis, and so on. (4) Display of visual results: usually, visualization tools are used to display the data analysis results in graphs, charts, or interfaces, highlighting the value of data, making the data results easier to communicate, more vivid and friendly, and more intuitive to feel the key information conveyed by the research results.

### 3.2. User Perception Analysis of Data Mining Based on Artificial Intelligence

The narrative of cultural and creative products emphasizes “theme,” focusing on the association and development of themes and subtopics. At the same time, designers are required to take into account both product and cultural aspects when conducting design analysis and be able to analyze the compatibility between narrative subtopics and design carriers. There are two ways to narrate cultural and creative products: (i) Determine the carrier of product design, such as whether the designed product is a brooch, folding fan, or bookmark, and then determine the narrative theme of this design. For example, the brooch is intended to express Miao culture, and Miao culture is the narrative theme of this design. (ii) Specify the narrative subtopic, and then find the product carrier suitable to reflect the subtopic. Finally, the designer extracts the cultural symbol elements from the narrative subtopic for design and creation. On the basis of the existing narrative design theory, this study further separates narrative subtopics into two directions, namely, image subtopics and cultural subtopics, as shown in Figure 1.

The article "Design Model of Cultural and Creative Products Using User Perception Demand Mining" was retracted in 2023. Reasons: suspected computer-generated content; unreliable results or conclusions; concerns about the data; concerns about the results or conclusions.

First, collect the cultural and image data that the theme can convey, then analyze the image subtopic and cultural subtopic under the narrative theme of cultural and creative products, and establish a narrative theme-narrative subtopic (including image subtopic and cultural image subtopic), the research idea of the design carrier. Then, the image subtopics that can represent the theme are selected by cluster analysis. Finally, the cultural subtopic and design are analyzed based on the perceptual image research method (optimized fuzzy comprehensive evaluation method). The determination of the image subtopic and the cultural subtopic will help the designer to grasp the overall design tone and enhance the cultural identity and recognizability of the product.

This paper introduces the main links of data mining, puts forward the main process of text data mining based on online comments, and briefly expounds the application tools of classification technology and clustering technology in text data mining. The development trend of industrial design puts forward the perceptual design method of products driven by artificial intelligence: (1) sort out the research status of users' perceptual cognition; (2) combined with computer science and users' perceptual cognitive characteristics, an efficient design method that can meet users' psychological needs is put forward, so as to enhance product competitiveness. As important text data, online reviews contain a lot of potential practical application value. Text mining technology can reveal the rich hidden information in the review content, such as review topics, product features, and user satisfaction.  Figure 2 shows the text data mining process with online comments as the data source.

Through the design process, we can closely grasp the user's perceptual cognition and turn it into the user's psychological needs, thus improving the user's satisfaction with the design works. In this design process, the artificial intelligence calculation method has been used many times, which effectively improves the design efficiency. The flowchart of the artificial intelligence-driven product perceptual design method is shown in Figure 3.

The article "Design Model of Cultural and Creative Products Using User Perception Demand Mining" was retracted in 2023. Reasons: suspected computer-generated content; unreliable results or conclusions; concerns about the data; concerns about the results or conclusions.

For the narrative analysis of an example of a cultural and creative product, the narrative theme can be summarized as a set *P*, the related image subtopic set is marked as *P*_*k*_, the cultural subtopic set is marked as *P*_*c*_, and the narrative theme *P* is expressed in the form of a divergent tree as follows:

(1) $$\begin{array}{c} P=\text{Tree}\left(P_{k},P_{c}\right),k=1,2,\ldots ,n;c=1,2,\ldots ,n. \end{array}$$

At the same time, under the application of this algorithm, if unknown sample data is added to the network in the subsequent error compensation process, the network can still correctly map from the input space to the output space. According to the various causes of errors in the spatial pattern analysis, a mathematical model is constructed:

(2) $$\begin{array}{c} O_{j}\left(t\right)=f\left(\left[\sum_{i=1}^{n}v_{ij}x_{i}\left(t-\tau_{ij}\right)\right]-T_{j}\right). \end{array}$$

### 3.3. Qualitative Analysis of Related Factors

In order to effectively reduce the influence of subjective thinking in the design decision-making process, cultural subtopics with a high degree of fit with the design carrier were selected. Fuzzy comprehensive evaluation is adopted here, the above-mentioned correlation evaluation factors are used as the evaluation basis for selecting cultural subtopics, the cumulative variance of the common factors in the above factor analysis is rotated, and the ratio of the rotated contribution rate to the corresponding variance percentage is used as the corresponding factor. The weights are used to select cultural subtopics. The specific process is as follows: First, define the set of perceptual comments *V*, *v* = (very important, important, general, unimportant, and very unimportant), and assign the value of perceptual comments by semantic difference method; that is, *v* = (5, 4, 3, 2, 1). Then, the set of relevance evaluation factors is set as *u*, and the expert evaluation method is used to evaluate each relevance evaluation factor to obtain the membership matrix *R*I, *R*2,…+, *RN* of the *n*th level index of relevance evaluation factors on the perceptual evaluation set *V*. Next, let the factor weight coefficient set be *W*, and perform fuzzy linear transformation on W to obtain fuzzy vector *B*:

(3) B=W·R=b,1  b,2…,bn.

Let the fuzzy comprehensive evaluation set of the I cultural subtopic be *B*_*i*_, *V*_*j*_ be the perceptual evaluation value corresponding to each evaluation value of *B*_*i*_(*b*_1_, *b*_2_,…, *b*_*i*_), and *G* be the comprehensive score; then

(4) G=∑ B·iVj∑Vj.

The article "Design Model of Cultural and Creative Products Using User Perception Demand Mining" was retracted in 2023. Reasons: suspected computer-generated content; unreliable results or conclusions; concerns about the data; concerns about the results or conclusions.

The multiple coefficient of determination is *R*^2^ in multiple linear regression; the total change in the dependent variable *Y*, the heavier the proportion of regression sum of squares (change),*R*^2^ The larger the value (usually between 0 and 1), and the stronger the fitting degree of the sample data, which means that the linear relationship between the independent variable and the dependent variable is closer; otherwise, it is more irrelevant. If it is equal to zero, it means that there is no relationship between the two parties. The multivariate linear regression model explained by the regression equation is expressed as follows:

(5) $$\begin{array}{c} R^{2}=\frac{\sum {\left(\overset{\wedge }{y}-\bar{y}\right)}^{2}}{\sum {\left(y-\bar{y}\right)}^{2}}=1-\frac{\left(y-y^{\wedge }\right)}{\left(y-y^{-}\right)}. \end{array}$$

Among them,

(6) $$\begin{array}{c} \left\{\begin{array}{c} \sum {\left(y-y^{\wedge }\right)}^{2}=\sum y^{2}-\left(b0\sum y+b_{1}\sum x1y+b_{2}\sum x2y+\cdots bk\sum xky\right),\\ \sum {\left(y-y^{-}\right)}^{2}=\sum y^{2}-\frac{1}{n}{\left(\sum y\right)}^{2}. \end{array}\right) \end{array}$$

The relationship between product modeling element domain *E* and user image domain *I* can be represented by matrix *B*:

(7) $$\begin{array}{c} B=E\cdot 1=\left[\begin{array}{c} E_{11}E_{12}\cdots E_{1m}\\ E_{21}E_{22}\cdots E_{2m}\\ ...\\ E_{n1}E_{n2}\cdots E_{nm} \end{array}\right]\times \left[\begin{array}{c} I_{1}\\ I_{2}\\ ...\\ I_{m} \end{array}\right]. \end{array}$$

Considering the different degrees of interaction between different elements, the importance coefficient should be added to the above formula. Let the importance coefficient between product modeling element domain *E* and user image domain *I* be matrix *T*, the importance coefficient between user feature domain and user image domain be matrix *W*, and the importance coefficient between user feature domain and modeling element domain be matrix *X*. The above formula can be rewritten as follows:

(8) $$\begin{array}{c} B^{\prime }=E\cdot I\cdot T,\\ C^{\prime }=U\cdot I\cdot W,\\ D^{\prime }=U\cdot E\cdot X. \end{array}$$

From another point of view, *D*′ actually reflects the relationship between *B*′ and *C*′, so it can be deduced that, for a specific user group, *X* is a function of *T* and *W*.

(9) $$\begin{array}{c} X=f\left(T,W\right). \end{array}$$

The original data is assigned a corresponding grade according to its average descending position in the overall data. In practical application, the connection between variables is irrelevant, so *p* can be calculated through simple steps. The difference between the grades of the two observed variables *d*_*i*_=*x*_*i*_ − *y*_*i*_; then, *p* is

(10) $$\begin{array}{c} \rho =1-\frac{6\sum d_{i}^{2}}{n\left(n^{2}-1\right)}. \end{array}$$

If RBF kernel function is used,

(11) $$\begin{array}{c} K\left(x_{C}i,X\right)=\exp\left(-\gamma {\left\|x_{i}-x\right\|}^{2}\right). \end{array}$$

After setting the training set and test set of the support vector machine, select the C-SVC mode in LIbsvm to model the support vector machine. Selecting RBF as the kernel function, the establishment of the model needs to find the optimal parameters *C* and *g* (i.e., *y*). A pattern recognition method based on statistical learning theory is proposed by a support vector machine. The research methods of perceptual images are summarized, respectively, including the method of screening original data, the method of acquiring perceptual images, the method of data processing and dimensionality reduction, and the method of dealing with the relationship between perceptual words and other variables. This method is simply described and illustrated. By using the K-CV cross-validation method to optimize the parameters, the parameter combination with the highest classification accuracy can be found.

The article "Design Model of Cultural and Creative Products Using User Perception Demand Mining" was retracted in 2023. Reasons: suspected computer-generated content; unreliable results or conclusions; concerns about the data; concerns about the results or conclusions.

## 4. Result Analysis and Discussion

The teapot, a representation of traditional Chinese culture, is significant from many perspectives, including traditional craftsmanship, regional cultural heritage, and cultural heritage. The teapot has established a separate craft system through the use of its traditional craftsmanship, and thanks to its distinctive national aesthetic and artistic features, it has gradually transformed from a utilitarian object into a collectible work of art. It also plays a crucial role in the technical aspects of Chinese traditional ceramics production. A nation or region's culture is a comprehensive reflection of its customs, traditional customs, lifestyles, ways of thinking, and values. Culture is defined as the sum of material wealth and spiritual wealth created in the process of human social development. Accordingly, research on Zisha teapots can not only analyze social and cultural phenomena in the Yixing region but also explore its research value in the areas of technology, sociology, economics, and so on and play a positive role in promoting the development and innovation of Yixing Zisha. This opens up a new research avenue for promoting traditional Chinese culture and regional cultural inheritance and protection. This study focuses on how subjects value subjective beauty, subjective image, and visual attention. The samples with decorative patterns on their surfaces and other comparable samples were removed to ensure the accuracy of the follow-up experiment, and the samples of the purple sand teapot that had been collected were then categorized and screened. Ball, Shiladle, Sifang, and ball jugs underwent multiple scale analysis and cluster analysis. Experimental samples included five different kinds of geometric-shaped purple clay pots, as seen in Figure 4.

The article "Design Model of Cultural and Creative Products Using User Perception Demand Mining" was retracted in 2023. Reasons: suspected computer-generated content; unreliable results or conclusions; concerns about the data; concerns about the results or conclusions.

The area of interest (AOI) in an eye movement experiment is used to frame a particular area and collect and analyze data from various eye-tracking indicators in the area, making the research more precise and focused. The division of the AOI area allows for the maximum elimination of other visual interferences while still obtaining intuitive data for each research object. According to the research goal of the eye movement experiment, which may be a single object or a specific area, the AOI area should be divided. Visual attention index data, visual search index data, and other index data are roughly the three categories into which the quantitative data in eye-tracking index data can be divided. In order to choose the eye movement index data that best meet the needs of the research for analysis, it is necessary to first screen the existing eye movement tracking data. Eye-tracking experiments will generate a significant amount of relevant eye movement data. In this study, we chose among the eye-tracking indicators the data of gaze time, number of gaze points, first gaze time, saccade time, times of retrospection, and gaze sequence, computed the average gaze time and the proportion of gaze time, and performed preliminary statistics. The statistical results are shown in Figure 5.

Descriptive analysis was performed on the eye-tracking data in the information area, and the statistical results are shown in Table 1.

From the task level, the design of cultural and creative products related to purple clay teapot can start from the tea drinking methods in different periods, explore the relationship between different tea drinking methods and corresponding tea set combinations, further extend to various tea activities and tea drinking customs such as tea art and tea ceremony, extract the modern tea cultural forms and cultural characteristics, and design relevant cultural and creative products in combination with the preferences of modern consumers.

The aforementioned data indicate that more than 80% of consumers place a high value on the novelty and cultural significance of Wenchuang products. Consumers are also worried about the product's usefulness, the designer, the product's origin story, the price, and the product's aesthetic quality. In contrast, the brand has little impact on consumer purchases. The connotation of cultural and creative products comes from their cultural value, which is distinct from that of other everyday necessities. The product itself incorporates the spiritual and emotional value of the cultural and creative content in addition to having certain practical and functional values. Innovatively incorporating cultural content into products that are both useful and culturally significant is the true definition of cultural and creative products. Additionally, as shown in Figure 6, the ever-richer living resources enable them to pay attention to the meaning behind more products, satisfy their needs for self-identity and literacy performance, and present more demanding product specifications.

The article "Design Model of Cultural and Creative Products Using User Perception Demand Mining" was retracted in 2023. Reasons: suspected computer-generated content; unreliable results or conclusions; concerns about the data; concerns about the results or conclusions.

Based on the theory of user sensibility, the above combs and analyzes the evolution history of purple sand teapot and its cultural ergonomic situation, interprets and excavates its cultural and design features, and summarizes three levels of cultural and creative product design related to purple sand teapot. At the same time, the subjective preference and visual preference of the overall shape of the purple clay teapot are studied by using the perceptual engineering method and eye-tracking technology, and the user's subjective image preference and subjective beauty preference are summarized to be applied to the design of cultural and creative products related to the purple clay teapot. From the user's point of view, the cultural points of Zisha teapot focus on the external expression of cultural temperament of Zisha teapot, and through the changes of details such as shape, material, and surface ornamentation, it reflects its connection with literati classes in different historical periods. From the tool level, the design of cultural and creative products can start with the relationship between ethnic groups and utensil shapes in different periods, aiming at a specific historical period, to study the lifestyle and excavate the cultural characteristics. Based on the analysis of the design attributes of cultural and creative products in this study, sketches were drawn for the product shape of the teapot, the shapes of various modeling elements were scrutinized and compared, and a plan was finally determined with reference to the opinions of the instructor and a number of subjects. Perform modeling refinement, modeling rendering, and final rendering, as shown in Figure 7.

According to FKQ's further investigation, the statistical results of cultural image characteristics of teapots are classified. The statistical results of FKQ's investigation are classified into five categories: attractive demand, expected demand, undifferentiated demand, reverse demand, and necessary demand. Then explore the real demands of users, and the final statistical calculation results are shown in Table 2.

The article "Design Model of Cultural and Creative Products Using User Perception Demand Mining" was retracted in 2023. Reasons: suspected computer-generated content; unreliable results or conclusions; concerns about the data; concerns about the results or conclusions.

According to statistics, A1 purple sand teapot color, A3 purple sand teapot shape, A7 teapot cultural experience form, and A12 emotional resonance in the design pattern of Chinese creative products belong to attractive demand. When these four kinds of factors are outstanding, they can greatly affect users' satisfaction. The other eight kinds of cultural image attributes show no difference demand, and such images have no strong correlation with users' satisfaction. Therefore, in order to embody the cultural elements of purple sand teapots in the process of creative design, we should focus on the charm demand and discuss the teapot color, traditional teapot shape, cultural experience form, and the application of emotional resonance in products, so as to improve the customer satisfaction of products, as shown in Figure 8.

In this study, the construction of the perceptual image space of the purple clay teapot is to quantify the fuzzy and difficult to express psychological feelings brought by the purple clay teapot to consumers through effective statistical and analytical means so as to obtain the basic data reflecting the relationship between the morphological elements of the purple clay teapot and the perceptual image and analyze the relationship between them and build a relationship model. Finally, the emotional image of consumers' uncertainty about the purple clay teapot is transformed into a specific design form. Finally, through expert evaluation, 10 pairs of perceptual words that best describe the overall appearance of the purple clay teapot are selected to be used in the design of the subjective image evaluation questionnaire of the purple clay teapot, as shown in Table 3.

The seven-order Likert scale was used to analyze the users' descriptions of the appearance and shape of purple sand teapots using the ten groups of perceptual word pairs that were previously identified, along with sample images of purple sand teapots. A positive number corresponds to the adjective on the right side of the midpoint “0,” while a negative number corresponds to the adjective on the left. The subject should select a score close to or equal to “3” if they believe that the overall modeling image of a particular purple sand teapot is more closely related to the right side adjective. The subject should select a score close to or equal to “−3” if they judge the purple sand teapot's overall modeling image as more closely resembling the adjective on the left. Through software interaction, the entire design process is completed, which conforms to the designer's way of thinking and operating habits, avoids the drawback that many design works cannot meet the needs of users, and offers designers effective, individualized software for product design assistance.

The article "Design Model of Cultural and Creative Products Using User Perception Demand Mining" was retracted in 2023. Reasons: suspected computer-generated content; unreliable results or conclusions; concerns about the data; concerns about the results or conclusions.

## 5. Conclusions

In this paper, I investigate the product perceptual design method and the user's perceptual cognition, and I propose an artificial intelligence-driven product perceptual design approach. The design of the optometer is used to confirm it, and it is determined that the method of design is workable and efficient. The purple clay teapot is used as the research subject for cultural and creative product design. The cultural characteristics of the purple clay teapot are extracted using the cultural ergonomics theory, and the users' preferences for the teapot's overall shape are studied using perceptual engineering and eye-tracking technology. This allows the authors to propose a cultural and creative product design strategy based on the cultural ergonomics situation. By using the perceptual engineering method, the perceptual image vocabulary is compiled, and a subjective questionnaire survey is used to gather user evaluation data on the overall design and various modeling components of the purple sand teapot. The quantitative analysis of the survey data is done using a statistical method, and the results show what users think about the general shape of the purple sand teapot in terms of subjective beauty and image preference. Finally, in order to direct the design of Wenchuang products, the cultural ergonomics context of the Zisha teapot is combined with the research findings regarding users' subjective preferences. The simulation results demonstrate that the algorithm used in this paper has an accuracy that is, on average, 9.34 percent greater than that of the data mining algorithm. Excavate the cultural design factors that meet user demands in order to provide a reference for businesses to design cultural and creative products that meet user needs. This result fully demonstrates that the proposed method for building volume optimization based on neural network and genetic algorithm can effectively reduce the time consumption required to run the program without affecting the algorithm's performance. In conclusion, the modern design utilizes the user's perceptual needs as a key design factor. Users' perceptual cognition can be accurately measured and design data transformed by combining perceptual engineering and artificial intelligence.

## Figures and Tables

**Figure 1:** Creative product narrative analysis ideas.

**Figure 2:** Data mining flowchart.

**Figure 3:** Flowchart of perceptual design method of artificial intelligence-driven products.

The article "Design Model of Cultural and Creative Products Using User Perception Demand Mining" was retracted in 2023. Reasons: suspected computer-generated content; unreliable results or conclusions; concerns about the data; concerns about the results or conclusions.

**Figure 4:** Zisha teapot sample. (a) Ball pot. (b) Shipiaohu. (c) Sifanghu. (d) Round pot. (e) Straight pot.

**Figure 5:** Statistics of the number of retrospectives in the eye-tracking experiment of the Zisha teapot.

**Figure 6:** Factors that consumers pay attention to when purchasing cultural and creative products.

**Figure 7:** Standardization coefficient.

**Figure 8:** Analysis of modeling data of purple clay pot.

**Table 1:** Descriptive analysis of eye-tracking data for each shape element of Zisha teapot.

Modeling elements (AOI)	Aoi1 pot twist	Aoi2 lid	Aoi3 handle	Aoi4 pot body	Aoi5 pot bottom	Aoi6 spout
Fixation time	915.555	1585.5584	1054.551	2685.455	345.425	815.512
Fixation points	2.454	3.845	5.4525	9.412	1.852	2.8863
Average fixation	368.455	345.1456	245.5785	286.586	200.084	378.4545
Time/ms	37.465	30.555	22.874	19.782	3.9	12.856
Fixation time	13.0	2.05	11.0	13.25	18.3	30.8
Specific gravity/%	2.1	3.0	2.5	9.8	1.5	2.8
First gaze	384.456	298.455	256.133	213.553	210.865	276.432
Saccade time	105.565	200.54	342.41556	256.8585	312.485	358.15
Look back times	0.5146	0.8546	0.440	0.3521	0.292	0.198
Gaze sequence	3.65	3.745	4.5465	2.275	5.982	3.785

**Table 2:** Fuzzy Kanon statistical results.

Evaluating indicator	A	M	O	I	R	Q	Category
A1	40	0	16	23	0	0	A
A2	32	2	22	38	0	0	I
A3	31	3	0	45	0	0	A
A4	30	0	12	26	0	0	I
A5	24	8	15	38	0	0	I
A6	12	10	21	44	0	0	I
A7	25	12	26	46	0	0	A
A8	28	5	0	38	0	0	I
A9	30	6	2	40	0	0	I
A10	24	11	8	18	0	0	I
A11	29	9	13	10	0	0	I
A12	18	10	0	48	0	0	A

**Table 3:** Final perceptual vocabulary pairs.

Serial number	Perceptual word pairs
1	Simple-complex
2	Refined-rough
3	Static-dynamic
4	Geometric-organic
5	Modern-classical
6	Individualized-ordinary
7	Lightweight-heavy
8	Soft-tough
9	Introverted-flamboyant
10	Elegant-simple

## Data Availability

The data used to support the findings of this study are available from the corresponding author upon request.
